# Investigation of three potential autoantibodies in Sjogren's syndrome and associated MALT lymphoma

**DOI:** 10.18632/oncotarget.15613

**Published:** 2017-02-22

**Authors:** Li Cui, Naseim Elzakra, Shuaimei Xu, Gary Guishan Xiao, Yan Yang, Shen Hu

**Affiliations:** ^1^ UCLA School of Dentistry, Los Angeles, CA 90095, USA; ^2^ UCLA Jonsson Comprehensive Cancer Center, Los Angeles, CA 900953, USA; ^3^ Department of Dentistry, Maoming People's Hospital, Maoming 525000, China; ^4^ Guangdong Provincial Stomatological Hospital, Guangzhou 510000, China; ^5^ School of Pharmaceutical Science and Technology, Dalian University of Technology, Dalian, 116024 China; ^6^ Department of Stomatology, Zhongnan Hospital, Wuhan University, Wuhan 430071, China

**Keywords:** Rho GDP-dissociation inhibitor 2, alpha-enolase, cofilin-1, primary Sjögren's syndrome, mucosal-associated lymphoid tissue lymphoma

## Abstract

Primary Sjögren's syndrome (pSS) is a chronic autoimmune disease which might progress to mucosal-associated lymphoid tissue lymphoma (pSS/MALT). Diagnosis of pSS requires an invasive tissue biopsy and a delay in diagnosis of pSS has been frequently reported. In this study, four proteins including cofilin-1, alpha-enolase, annexin A2 and Rho GDP-dissociation inhibitor 2 (RGI2) were found to be over-expressed in pSS and pSS/MALT by 2D gel electrophoresis/mass spectrometry, and the finding was verified by the microarray analysis and western blotting results. We then developed enzyme-linked immunosorbent assays for autoantibodies including anti-cofilin-1, anti-alpha-enolase and anti-RGI2 with good *quantitative* ability. The expression levels of salivary anti-cofilin-1, anti-alpha-enolase and anti-RGI2 were found to be the highest in pSS/MALT patients and lowest in healthy controls. The combination of these three antiantibodies yielded an “area under the curve” (AUC) value of 0.94 with an 86% sensitivity and 93% specificity in distinguishing patients with pSS from healthy controls, an AUC value of 0.99 with a 95% sensitivity and 94% specificity in distinguishing patients with pSS/MALT from healthy controls and an AUC value of 0.86 with a 75% sensitivity and 94% specificity in distinguishing pSS/MALT patients from pSS patients. Collectively, we have successfully identified a panel of potential autoantigens that are progressively up-regulated during the development of pSS and its progression to MALT lymphoma. The autoantibody biomarkers may be used to help diagnose pSS and predict its progression to MALT lymphoma.

## INTRODUCTION

Primary Sjögren's syndrome (pSS) is a chronic disorder of unknown cause marked by dry eye/dry mouth symptoms as a result of an autoimmune attack on the salivary and lacrimal glands. Injury, viruses, and/or self-antigens might be the potential stimulus driving the initiation and progression of this autoimmune disease [1, 2]. The common histopathological feature of all organs affected by pSS is a potentially progressive lymphocytic infiltration. The predominant cell type infiltrating the gland tissues is T cells, and the number of CD4+ T cells is bout 3-5 times more than that of CD8+ T cells. B cells and natural killer cells constitute approximately 20% and 5% of the total infiltrating population respectively [3–4]. The percentage of B cell increased in the advanced cases of pSS and persistent B cell activation might enhance the risk of the progression of pSS to mucosa-associated lymphoid tissue (MALT) lymphomas (pSS/MALT) [5–6].

Saliva is produced by three pairs of major salivary glands (the parotid, submandibular and sublingual glands) and numerous minor ones. It has been demonstrated that saliva contains many informative molecules that can be useful for diagnosing human diseases such as HIV, cancer, cardiovascular diseases and diabetes [7–10]. In recent years, saliva has attracted widespread interest as a diagnostic medium for simple and rapid disease testing. The advantages of using saliva for disease diagnostics include ease of access, noninvasive sample collection, increased acceptance by patients, and reduced risks of infectious disease transmission [11, 12]. Since salivary glands are the major target organs of pSS and pSS/MALT lymphoma, identifying the changes in gene and protein expression in saliva might not only help discover biomarkers for pSS or pSS/MALT lymphoma, but also contribute to the understanding of the molecular mechanisms underlying pSS and its development into MALT lymphoma.

Although continuous efforts have been made to search saliva biomarkers for pSS, currently no clinically validated biomarker is available to predict the progression of pSS to pSS/MALT lymphoma. In this study, we have identified a number of significantly over-expressed proteins in the salivary gland tissues of patients with pSS or pSS/MALT lymphoma using 2-D gel electrophoresis (2-DGE) with mass spectrometry (MS). A panel of these proteins, including cofilin-1, alpha-enolase and Rho GDP-dissociation inhibitor 2 (RGI2), were further verified and the levels of saliva autoantibodies to these proteins were also measured. Our results indicate that these autoantibodies may serve as biomarkers for pSS and its progression to pSS/MALT lymphoma with high specificity and sensitivity.

## RESULTS

### 2-DGE/MS analysis of proteins in the parotid gland tissues of pSS and pSS/MALT lymphoma

Figure 1 shows 2-DGE separation of the parotid gland tissue proteins of pSS, pSS/MALT and non-SS control. The proteins that are up-regulated (>1.5 fold) in pSS patients (vs non-SS control) are listed in Table 1. Similarly, the proteins that are over-expressed (>1.5 fold) in pSS/MALT patients when compared to both pSS and control samples are listed in Table 2.

**Figure 1:** 2-DGE of the proteins in salivary gland tissues from non-SS controls and patients with pSS or pSS/MALT lymphoma Equal amount of proteins were pooled from the 6 individuals in each group (control, pSS & pSS/MALT) and mapped out using the IPG strips (pI 3-10 NL) and 8-16% PAGE gels.

**Table 1:** Salivary gland tissue proteins over-expressed (>1.5 fold) in pSS patients when compared to control subjects

Accession#	M.W./pI	Protein name
IPI00021536.1	15921.4/4.15	Calmodulin-like protein 5
IPI00181833.3	66861.6/7.91	Epidermal growth factor receptor kinase substrate 8-like protein 3
IPI00007425.1	93835.4/5.21	Desmocollin 1b
IPI00025753.1	113715.8/4.76	Desmoglein-1
IPI00788705.1	30319.7/6.10	JUP 30kDa protein
IPI00654788.1	133604.8/10.0	Profilaggrin
IPI00003817.3	22988.8/4.94	Rho GDP-dissociation inhibitor 2
IPI00021841.1	30778.6/5.46	Apolipoprotein A-I
IPI00215983.3	28871.0/6.67	Carbonic anhydrase 1
IPI00373937.2	60541.4/6.52	Suprabasin
IPI00012011.6	18503.4/8.19	Cofilin-1
IPI00027350.3	21892.8/5.59	Peroxiredoxin-2
IPI00219953.5	25855.7/7.96	Cytidylate kinase
IPI00171438.2	47629.5/5.58	Thioredoxin domain-containing protein 5
IPI00465436.4	59756.7/6.97	Catalase
IPI00016801.1	61398.5/7.68	Glutamate dehydrogenase 1, mitochondrial
IPI00027146.1	61434.6/8.57	Glutamate dehydrogenase 2, mitochondrial
IPI00473031.6	39855.3/8.21	Alcohol dehydrogenase 1B
IPI00465248.5	47169.6/7.16	Alpha-enolase
IPI00027547.2	11284.8/6.12	Dermcidin
IPI00291006.1	35532.1/8.79	Malate dehydrogenase, mitochondrial
IPI00847322.1	24751.0/8.38	Superoxide dismutase
IPI00007002.3	52000.0/8.85	AarF domain containing kinase 1
IPI00418169.3	40411.9/8.50	Annexin A2
IPI00290158.6	77702.8/9.96	Serine/threonine-protein kinase MARK2
IPI00472610.2	52667.3/7.39	IGHM protein
IPI00426051.3	51099.5/7.55	Rheumatoid factor RF-IP15

**Table 2:** Salivary gland tissue proteins over-expressed (>1.5 fold) in pSS/MALT compared to pSS and control subjects

Accession#	M.W./pI	Protein Name
IPI00296441.5	40765.2/5.57	Adenosine deaminase
IPI00027341.1	38518.3/5.85	CAPG Macrophage-capping protein
IPI00848090.1	38499.3/5.79	CAPG gelsolin-like capping protein
IPI00017704.3	15945.9/5.38	Coactosin-like protein
IPI00007926.1	19109.3/4.82	c-Myc-responsive protein Rcl
IPI00003817.3	22988.8/4.94	Rho GDP-dissociation inhibitor 2
IPI00178083.2	29079.6/4.60	Tropomyosin alpha-3 chain
IPI00010779.4	28522.6/4.52	Tropomyosin alpha-4 chain
IPI00010896.3	26923.6/4.94	Chloride intracellular channel protein 1
IPI00292812.6	46488.7/4.74	Protein TMED8
IPI00642256.1	29296.1/6.51	Capping protein muscle Z-line, beta
IPI00026185.5	31351.3/5.24	F-actin-capping protein subunit beta
IPI00032575.3	34794.2/5.29	Glyoxalase domain-containing protein 4
IPI00060715.1	35701.5/5.36	BTB/POZ domain-containing protein KCTD12
IPI00465248.5	47169.6/7.16	Alpha-enolase
IPI00397801.4	248071.8/8.09	Ifapsoriasin
IPI00027341.1	38518.3/5.85	Macrophage-capping protein
IPI00013894.1	62639.9/6.39	Stress-induced-phosphoprotein 1
IPI00419585.9	18013.4/7.82	Peptidyl-prolyl cis-trans isomerase A
IPI00169383.3	44615.4/8.12	Phosphoglycerate kinase 1
IPI00219568.4	44796.9/8.69	Phosphoglycerate kinase 2
IPI00219806.6	11457.9/6.34	Protein S100-A7
IPI00418169.3	40411.9/8.50	Annexin A2
IPI00000874.1	22111.2/8.21	Peroxiredoxin-1
IPI00012011.6	18503.4/8.19	Cofilin-1
IPI00413344.3	18737.5/8.12	Cofilin-2
IPI00010154.3	50583.4/4.86	Rab GDP dissociation inhibitor alpha
IPI00021327.3	25207.2/5.87	Growth factor receptor-bound protein 2
IPI00014424.1	50470.8/9.36	Elongation factor 1-alpha 2
IPI00396485.3	50141.5/9.35	Elongation factor 1-alpha 1

### Verification of a panel of target proteins identified by 2-DGE/MS

Among the significantly up-regulated proteins in pSS/MALT, we validated four proteins including cofilin-1, alpha-enolase, annexin A2 and RGI2, using western blotting. They were most significantly over-expressed in pSS/MALT while most under-expressed in the controls (Figure 2). The western blotting results not only further corroborated our initial finding, but also suggested that these proteins were progressively up-regulated during the progression of pSS to pSS/MALT. Our previous microarray study also indicated that the gene expression levels of these proteins were over-expressed in pSS [13]. The relative expression levels of cofilin-1, alpha-enolase, annexin A2 and RGI2 in pSS patients were higher than those in controls. However, their levels were lower in pSS patients when compared to patients with pSS/MALT (Table 3).

**Figure 2:** Western blot analysis of cofilin-1, alpha-enolase, annexin A2 and RGI2 in salivary gland tissues from non-SS controls (n=6) to patients with pSS (n=6) or pSS/MALT lymphoma (n=6) The results indicated that the expression levels of the four proteins were highest in MALT lymphoma while lowest in non-SS controls.

**Table 3:** Differential expression of cofilin-1, alpha-enolase, annexin A2 and RGI2 in salivary gland tissues among pSS/MALT, pSS and control subjects as revealed by DNA microarray analysis

pSS vs control			pSS/MALT vs pSS		
Gene symbol	Fold changes	P	Gene symbol	Fold changes	P
Cofilin-1	1.42	3.54e-6	Cofilin-1	1.33	0.035
Alpha-enolase	1.19	0.018	Alpha-enolase	1.64	0.008
Annexin A2	1.16	0.012	Annexin A2	1.24	0.141
RGI2	5.36	7.87e-6	RGI2	2.15	2.02e-6

### Development of ELISAs for anti-coffilin-1, anti-alpha-enolase, anti-RGI2

Since commercial ELISA kits for anti-cofilin-1, anti-alpha-enolase, and anti-RGI2 were not available, home-made ELISAs were developed for saliva testing of these autoantibodies. We used an equally pooled saliva sample from 10 patients with pSS to establish calibration curves, with an assumption that the concentration of these antiantibodies (anti-cofilin-1, anti-alpha-enolase and anti-RGI2) was 300 Units/ml in the pooled sample. In fact, commercial ELISA kits for autoantibodies use reference serum for establishing the calibration curves. Figure 3 presents the calibration curves for the three antiantibodies established from a serial dilution of the pooled saliva sample with antiantibodies concentrations of 300, 120, 48, 19.2,7.68, 3.071 and 0 Units/ml. The assays are quantitative for anti-cofilin-1(y=0.0009x+0.0281, R^2^=0.9973), anti-alpha-enolase (y=0.0012x+0.0041, R^2^=0.9890), and anti-RGI2 (y=0.0014x+0.0028, R^2^=0.9986).

**Figure 3:** Calibration curves of the ELISAs for anti-coffilin-1, anti-alpha-enolase and anti-RGI2

### ELISA of the three autoantibody biomarkers in saliva samples

We then measured the three autoantibody biomarkers in saliva samples from 50 pSS patients, 20 pSS/MALT patients and 50 healthy control subjects. Figure 4 showed the expression levels of the three autoantibody biomarkers (anti-coffilin-1, anti-alpha-enolase, anti-RGI2) were all over-expressed in pSS/MALT patients compared with both pSS patients and healthy control subjects (P<0.01; P<0.001). Their levels were significantly higher in the saliva samples of pSS patients compared to those from healthy subjects (P<0.01; P<0.001). These data clearly demonstrated that the patients with pSS and pSS/MALT lymphoma had significant over-expression of cofilin-1, alpha-enolase and Rho GDI2 as well as their respective antiantibodies.

**Figure 4:** ELISA quantification of three potential saliva autoantibody biomarkers on a new patient/control cohort (n=50 for pSS, n=20 for pSS/MALT and n=50 for control) The result showed that the salivary levels of these potential autoantibodies were highest in pSS/MALT while lowest in the healthy controls (**P<0.01; ***P<0.001)

### The potential clinical utility of the three autoantibody biomarkers for pSS and pSS/MALT

As shown in Figure 5, the ROC analysis was performed to evaluate pre-clinical utility of these potential biomarkers and to assess if combining biomarkers may improve the sensitivity and specificity. The overall performance of the three potential biomarkers in distinguishing pSS, pSS/MALT and healthy subjects is summarized in Tables 4–6. For pSS versus control, the AUC values of anti-coffilin-1, anti-alpha-enolase, anti-RGI2 were 0.81, 0.82 and 0.85, respectively. For pSS/MALT vs control, the AUC values of anti-coffilin-1, anti-alpha-enolase, anti-RGI2 were 0.93, 0.93 and 0.94, respectively. For pSS/MALT vs pSS, the AUC values of anti-coffilin-1, anti-alpha-enolase, anti-RGI2 were 0.80, 0.78 and 0.74 for pSS/MALT, respectively.

**Figure 5:** Receiver operating characteristic (ROC) analysis of the three potential biomarkers (anti-cofilin-1, anti-alpha-enolase and anti-RGI2) for the detection of pSS or pSS/MALT

**Table 4:** Performance characteristics of the biomarkers for distinguishing pSS and healthy control subjects

Biomarker	AUC	Sensitivity	Specificity
Anti-cofilin-1	0.81	0.76	0.82
Anti-α-enolase	0.82	0.82	0.74
Anti-RGI2	0.85	0.84	0.74
Anti-cofilin-1+Anti-α-enolase+Anti-RGI2	0.94	0.86	0.93

**Table 5:** Performance characteristics of the biomarkers for distinguishing pSS/MALT and healthy control subjects

Biomarker	AUC	Sensitivity	Specificity
Anti-cofilin-1	0.93	0.80	0.90
Anti-α-enolase	0.93	0.90	0.84
Anti-RGI2	0.94	0.90	0.80
Anti-cofilin-1+Anti-α-enolase+Anti-RGI2	0.99	0.95	0.94

**Table 6:** Performance characteristics of the biomarkers for distinguishing pSS/MALT and pSS

Biomarker	AUC	Sensitivity	Specificity
Anti-cofilin-1	0.80	0.70	0.86
Anti-α-enolase	0.78	0.65	0.84
Anti-RGI2	0.74	0.50	0.92
Anti-cofilin-1+Anti-α-enolase+Anti-RGI2	0.86	0.75	0.94

The combination of these three antiantibodies yielded a better AUC value of 0.94 with an 86% sensitivity and 93% specificity in distinguishing patients with pSS from healthy control subjects and an AUC value of 0.99 with a 95% sensitivity and 94% specificity in distinguishing patients with pSS/MALT from healthy control subjects as well as an AUC value of 0.86 with a 75% sensitivity and 94% specificity in distinguishing patients with pSS/MALT from pSS patients (Figure 6).

**Figure 6:** The combination of three potential biomarkers (anti-cofilin-1, anti-alpha-enolase and anti-RGI2) improved the AUC values as well as sensitivity and specificity for the detection of pSS or pSS/MALT

## DISCUSSION

pSS remains a challenging public health problem worldwide because of its high prevalence and no cure for the disease. A number of autoantibodies have been reported in patients with pSS. These molecules produced by hyperactivated B cells can cause the destruction of exocrine glands, especially lacrimal and salivary glands, and also other external glands such as the pancreas, mucous glands of the gastrointestinal and respiratory tract or bile secretion. Studies have confirmed that there is an increased incidence of cancer especially lymphoma in patients with pSS [14, 15]. However, the pathogenesis of pSS as well as its development into MALT lymphoma remains reclusive.

Understanding of the molecular mechanism responsible for pSS and its progression to MALT lymphoma requires molecular analysis of the affected salivary gland tissues from the disease patients. In this study, we first profiled parotid gland tissue proteins from pSS, pSS/MALT and control subjects with 2-DGE/MS, and identified a number of new protein targets that might be associated with pathogenesis of pSS or pSS/MALT. We then demonstrated that cofilin-1, alpha-enolase, annexin A2 and RGI2 were most abundant in pSS/MALT at both protein and gene expression levels, which confirmed our 2-DGE/MS results. Among the proteins aberrantly expressed in pSS patients compared with the non-SS controls, some are functionally related to immune response, apoptosis, cell adhesion and anti-oxidation. As anticipated, rheumatoid factor RF-IP15 was up-regulated in pSS, although this was the only autoantibody revealed by the 2-DGE/MS approach. The antioxidant enzymes including superoxide dismutase and catalase were found to be increased in pSS patients. This is somewhat consistent with previous findings, which indicated that the antioxidant thioredoxin was overexpressed in pSS tissues [16]. We speculated that the upregulation of antioxidants is due to cellular response to protect the salivary glands of pSS patients from oxidative stress and tissue damage. Many proteins that are up-regulated in pSS/MALT lymphoma are mostly involved in signal transduction, gene regulation, immune response and oxidative stress. Cofilin-1 is a key molecule controlling actin dynamics by depolymerizing actin filaments. Autoantibodies directed against cofilin-1 have been found in patients suffering from autoimmune diseases such as rheumatoid arthritis, systemic lupus erythematosus, polymyositis, dermatomyositis, and Behçet's disease [17]. In addition, dysregulation of cofilin-1 has been associated with carcinogenesis [18]. Alpha-enolase is a multifunctional glycolytic enzyme that has been implicated in other autoimmune diseases such as Hashimoto's encephalopathy [19]. We previously also found that salivary alpha-enolase was significantly elevated in patients with pSS compared to both SLE patients and healthy controls [20]. Alpha-enolase can also promote carcinogenesis in various types of cancer including lymphoma, indicating it might play an important role in the progression of pSS into pSS/MALT lymphoma [21–23]. Annexin A2 is a pleiotropic protein that regulates diverse cellular processes [24, 25]. It was significantly up-regulated in a number of malignant tumors and also associated with drug resistance and poor prognosis [26, 27]. Our study added a new evidence about the role of Annexin A2 in transformation of lymphoma. RGI2 is known as a negative regulator of Rho family GTPase and preferentially expressed in hematopoietic cells [28]. Perturbation of RGI2 signaling is important for tumorigenesis while its role in cancer progression appears to depend on the tumor type [29, 30]. Upregulation of RGI2 has been found to induce epithelial-mesenchymal transition in cancer cells to promote invasion and metastasis [30]. Overexpression of these proteins in pSS and pSS/MALT lymphoma suggested that they are not only important for pathogenesis of pSS, but also, more importantly, might play a crucial role in the progression of pSS to pSS/MALT lymphoma

In order to minimize life altering complications such as total loss of glandular functions and possibly other damaged internal organs, early diagnosis is critical for providing appropriate treatment prior to aggressive stages of pSS. The development of autoantibodies has been observed in all autoimmune disorders including pSS and occurs years before the clinical symptoms of autoimmune diseases. Therefore, autoantibodies (e.g., anti-SSA and anti-SSB) appears to be very promising biomarker targets that can be used in clinics to help diagnose pSS. However, it is also well known that many of the autoantibodies are only positive in a fraction of patients with an autoimmune disease and also present in patients with other autoimmune diseases. To tackle this challenge, it often requires combining multiple autoantibody biomarkers so that the diagnostic assay can be more sensitive and specific for the disease detection.

Since no commercial ELISA kit is available for detecting the autoantibodies against cofilin-1, alpha-enolase or RGI2, we have developed respective ELISAs to quantify their levels in saliva samples of patients with pSS or pSS/MALT lymphoma. Consistent with our findings in the parotid tissues, the expression levels of anti-alpha-enolase, anti-cofilin-1 and anti-RGI2 were highest in the saliva samples of patients with pSS/MALT, while lowest in the saliva sample of healthy subjects. It is possible that upregulation of anti-alpha-enolase, anti-cofilin-1 and anti-RGI2 may promote the development of pSS and pSS/MALT lymphoma, but further studies are certainly warranted to elucidate the potential molecular mechanisms. Our studies have clearly indicated salivary anti-alpha-enolase, anti-cofilin-1 and anti-RGI2 may be combinatorily used for highly sensitive and specific detection of pSS and pSS/MALT. These biomarkers not only distinguish pSS patients or pSS/MALT patients from healthy controls but more importantly can also differentiate pSS/MALT from pSS patients, which may be useful to predict the progression of pSS to MALT lymphoma. Nevertheless, one shortcoming of using salivary biomarkers for diagnosis is that this approach may only apply to patients with residual salivary function. In addition, due to relatively low conversion rate of pSS to MALT lymphoma, we had limited samples size for the pSS/MALT study. Future large-scale validation studies are needed for further testing these potential salivary biomarkers on new patients with pSS or pSS/MALT lymphoma.

## MATERIALS AND METHODS

### Patient cohort

The study was approved by the Ethic Committee of the Zhongnan Hospital, Maoming People's Hospital and Guangdong Provincial Stomatological Hospital. Written informed consent was obtained from all the participants for the use of their tissue and saliva specimens. All pSS patients met diagnosis criteria according to the US-EU criteria. pSS/MALT patients were diagnosed based on the existence of extranodal MALT lymphoma with concomitant pSS. For the tissue samples, the parotid biopsies of pSS and pSS/MALT patients were taken under local anesthesia. Control parotid biopsies (residual normal parotid tissues) were obtained from patients with chronic obstructive parotitis received parotidectomy after failure of conservative treatment. As for the saliva sample analysis, all subjects enrolled were Han Chinese female. All the healthy control participants were negative for serum anti-SSA/SSB antibodies, and there were no sicca complaints including oral and ocular dryness.

### Saliva sample collection

Whole saliva collection was performed at the Maoming People's Hospital, Zhongnan Hospital and Affiliated Stomatology Hospital of Southern Medical University using our standardized saliva collection protocols. Subjects were asked to refrain from eating, drinking, smoking, or performing oral hygiene procedures for at least 1 h prior to saliva collection. Stimulated whole saliva was collected over a period of 15 minutes by chewing on paraffin wax. The saliva samples were processed immediately with addition of protease inhibitors (Sigma, St. Louis, MO) and then centrifuged at 2,600*g* for 15 minutes at 4°C. The supernatant was removed from the pellet, immediately aliquoted, and stored at -80°C [13].

### Tissue protein sample preparation

The PARIS™ kit (Ambion, Austin, TX) was used to extract proteins from snap-froze glandular tissues. The total protein amount of each tissue samples was measured using the 2-D Quant Kit (GE Healthcare, Piscataway, NJ). Each sample was then purified with 2-D Cleanup Kit (GE Healthcare), and re-dissolved in rehydration buffer. Due to the limited amount of the tissues, the samples from the controls, pSS or pSS/MALT patients (n=6) were pooled, respectively, at equal amounts for the 2-DGE analysis.

### 2-DGE analysis and protein identification

Approximately 300-μg proteins from each pooled samples were used for 2-DGE analysis. 2-DGE was performed using the Immobilized pH gradient (IPG) gel strips (17cm, pI 3-10 NL) for IEF and 8-16% pre-cast gels for SDS-PAGE (Bio-Rad). After staining with Sypro Ruby, the gels were scanned and analyzed using the PDQuest program (Bio-Rad). The proteins spots showing over 1.5 fold changes were excised for in-gel tryptic digestion, and the resulting peptides were analyzed by LC-MS/MS (Eksigent Nano-LC & Thermo LTQ), as previously described [31]. Database searching was performed against the International Protein Index (IPI) human proteome database using the SEQUEST search engine (Thermo Scientific).

### Western blotting

Protein samples were separated with a 4-12% Bis-Tris NuPAGE gel (Invitrogen) and transferred onto nitrocellulose membrane by Trans-blot SD semi-dry transfer cell (Bio-Rad). After saturating with 5% milk in Tris Buffered Saline-Tween (TBST) buffer, the membranes were sequentially incubated with primary antibodies (Santa Cruz Biotech) overnight at 4°C and HRP-linked secondary antibodies, respectively (GE Healthcare). The detection was performed with the ECL-Plus Western blotting reagent kit (GE Healthcare).

### ELISA

ELISA was developed to measure anti-coffilin-1, anti-alpha-enolase, anti-RGI2 levels in the saliva samples of pSS/MALT, pSS and healthy control patients. To coat the plate, a human recombinant protein (cofilin: Cytoskeleton Inc; alpha-enolase and RGI2: Mybiosource Inc) were diluted in 100mM sodium bicarbonate/carbonate buffer at a concentration of 2ug/ml, followed by the addition of 100μl into each well. The proteins were allowed to bind to the wells overnight at 4°C. The next day the coating solution was removed and the plate was washed four times with approximately 300 μl of TBST washing buffer (1x). The coated wells were blocked by adding 250μl blocking buffer (5% non-fat dry milk and 1% BSA in TBST) for 2 hours. The plate was then washed three times with the same wash buffer. Calibration curves were established by using an equally pooled (n=10) saliva sample from pSS patients, assuming the concentration is 300U/mL. A serial of dilution of the pooled sample was then performed to form concentrations of 300, 120, 48, 19.2,7.68, and 3.072 U/ml. To measure the autoantibody, samples were diluted in sample buffer (1x TBST) and loaded in duplicate, onto a 96 microwell plate coated with human recombinant protein. After incubation for 1 hour on a shaker, the microwell strips were washed four times with approximately 300 μl of washing buffer (1x TBST), followed by the addition of 100 μl of enzyme conjugate reagent (Rabbit anti-human IgG, HRP) to each well. The plate was incubated again for 30 minutes followed by 4 times washing with the washing buffer. Subsequently, 100 μl of TMB solution was added to each wells and incubated in the dark for 10 minutes. Finally, stop solution (100 μl) was added to each well and the absorbance was measured at 450 and 620 nm. The autoantibody levels were determined according to the calibration curves.

### Statistical analysis

Data analysis was performed with the GraphPad Prism and MedCalc software. The data were expressed as the mean ± standard deviation, and analyzed by the One Way ANOVA with post-hoc Tukey HSD test. For the microarray data analysis, we first extracted the original data from our previous study, and then compared the expression levels of cofilin-1, alpha-enolase, annexin A2 and RGI2 between two different groups. Receiver operating characteristic (ROC) analysis was used to estimate the performance of potential biomarkers and evaluate if combining biomarkers improves sensitivity and specificity. P values<0.05 were regarded as statistically significant.
